# Alienation Control Technology of Information Pushed by Intelligent Algorithms in Media Communication

This article has been retracted.

**DOI:** 10.1155/2022/4855254

**Published:** 2022-06-27

**Authors:** Yang Cheng, Ming Cheng

**Affiliations:** School of Journalism and Communication, Wuhan University, Wuhan 430072, Hubei, China

## Abstract

“Information alienation” is a concept formed by combining the idea of “alienation” in philosophy with the characteristics of information itself. Information is a universal property of matter and an objectively existing form of material movement. The purpose of this paper is to study and analyze the alienation technology control of push information based on intelligent algorithms and describe the information alienation. This paper puts forward the problem of pushing information, which is based on intelligent algorithm, then elaborates around the concept of intelligent algorithm and related algorithms, and designs and analyzes the control of media information alienation. The experimental results show that, in the questionnaire survey, 72.34% of the people who very frequently swipe unfriendly information account for a very large proportion. People will always swipe it in various software applications, which is unavoidable. How to control the problem of information alienation needs to be controlled from the user level, the design media level, and the government level.

## 1. Introduction

In the information age, traditional media are declining day by day, and network media represented by Internet technology has become the main channel for information dissemination and circulation. The low threshold and interactivity of new media make the volume of information expand and the quality of information decline; the speed of information dissemination is getting faster and faster, and public opinion does not change in different media channels. In today's increasingly blurred boundaries between communicators and audiences, public noise has become a prominent feature of the Internet communication era. In the face of emergencies with the characteristics of suddenness, abnormality, destructiveness, and seriousness, media reports, government responses, and public opinion have become important factors affecting the direction of emergencies.

It is not surprising that users receive push notifications from websites, software clients, emails, and text messages through their mobile phones. However, people do not welcome this new thing with joy, especially under the negative influence of spam messages; users' acceptance of push messages has dropped sharply, resulting in mobile push messages failing to play its due commercial value. Therefore, in order to improve the acceptance of push information by Chinese users, it is necessary to analyze the influencing factors of users' acceptance of mobile push information.

The innovations of this paper are the following: (1) this paper combines intelligent algorithm with push information, introduces the theory and related methods of intelligent algorithm in detail, and mainly introduces simulated annealing algorithm, legacy algorithm, and ant colony algorithm. (2) In the face of push information, this paper investigates the frequency of people usually receiving dirty information and designs the push information model.

## 2. Related Work

Since the 1970s, with the development of bionics, genetics, and artificial intelligence, many scholars have begun to apply intelligent algorithms in the field of optimization to solve related problems. Zhao et al. propose an efficient method based on image segmentation and swarm intelligence (SI) algorithm with parameters used to detect each level through an invariable scale feature transformation scheme (SIFT). The experimental results demonstrate the good performance of the proposed method, which can effectively identify CMF images with small or smooth clonal regions. However, their experiments were less frequent [1]. Sheng et al. combine multiscale wavelet transform, particle swarm parameter optimization, and adaptive filtering algorithm improvement to obtain an applicable intelligent adaptive filtering algorithm. They simulated the algorithm and verified the actual engineering experimental data on the software platform, proving that the proposed algorithm is more suitable for practical engineering applications than the traditional adaptive filtering algorithm. However, its performance is lower [2]. Kim and Katipamula describe the development and validation of intelligent load control (ILC) algorithms for managing loads in buildings or groups of buildings using quantitative and qualitative criteria. By anticipating future demand, the process can be extended to add advanced controls to ease comfort while reducing RTU operation to manage peak demand. However, it consumes a lot of energy [3]. To bridge the time during GNSS outages, Zhang and Wang propose a novel hybrid intelligence algorithm that combines a discrete grey predictor (DGP) and a multilayer perceptron (MLP) neural network (DGP-MLP). To evaluate the effectiveness of the proposed method, they performed four GNSS outages on real field test data under different conditions. Experimental results show that the proposed method can significantly improve the positioning accuracy during GNSS outages. However, this process is more complicated [4]. Yang et al. proposed a theoretical extension of a novel intelligent algorithm Extended Support Vector Data Description (E-SVDD) for analyzing and controlling dynamic swarms for macroscopic and microscopic behavior prediction in automotive collision avoidance systems. The results confirm the improved performance and effectiveness of the proposed control logic. However, this data does not support the results well [5]. Nabih-Ali et al. propose an intelligent algorithm for heart disease diagnosis using phonocardiogram (PCG). The proposed technique consists of four stages: data acquisition, preprocessing, feature extraction, and classification. Finally, an artificial neural network (ANN) has been used in the classification stage with an overall accuracy of 97%. However, its application scope is limited [6]. Ding et al. deeply analyzed the method and experimental exploration of remote mobile medical information collection based on the Internet of Things and intelligent algorithms and successfully proved that the Internet of Things technology and intelligent algorithms have a certain positive significance for medical information collection and tracking upward medical services. The human telemedicine information collection system based on the Internet of Things and other related technologies can accurately and timely detect the patient's blood pressure, blood sugar, and other health data and then provide corresponding medical services. However, its usage conditions are demanding [7]. Yuan et al. use the face recognition method for identity authentication and use the improved elastic template matching algorithm to establish an intelligent classification method of dynamic face elastic model. Simulations show that the proposed method can intelligently adapt to various environments without reducing accuracy. However, it is less accurate [8].

## 3. Smart Way to Push Information

### 3.1. Media Communication

Communication media refers to information dissemination agencies, which can be private or official [9–11]. The rapidly growing concept of social media is vaguely defined but does not hinder its development. Today's social media comes in various forms and has unique characteristics that are different from traditional media [12].

Openness is the range of users participating in platform interactions. Before newspapers, magazines, etc., the requirements for manuscripts were very strict, and the content of each module was “professional,” which required all those involved in the production of traditional means to have certain professional qualities. The growth of the Internet limits user engagement, and social media makes up for that, with low restrictions on using social media and high levels of transparency.

Shareability: the huge user base makes the content covered on social media extremely extensive. With the development of Web 2.0, the state of user-generated content development (UGC) has gradually matured. According to different content formats, photos, music, videos, articles, etc. can be shared between users.

Interactivity: on social media, anyone can participate in topic interaction and information exchange in real time [13–15]. Participation limits are very low, regardless of the quality of the presentation and the professionalism of the topic. This form of two-way communication stimulates engagement, awareness, and information exchange among users. It greatly promotes the flow of information, expands the scope of information dissemination, and increases the output of information. As consumers (users), after realizing that they can only passively accept the pleasure of subjective choices, they are more willing to interact and communicate in a timely manner. This virtuous cycle has given a huge boost to the rapid growth of social media.

### 3.2. Alienation Technology of Push Information

“Information alienation” is a concept formed by combining the idea of “alienation” in philosophy with the characteristics of information itself. Information is the universal property of matter and the objective existence form of matter movement. Some scholars divide information into three categories: physical information, biological information, and social information. This paper studies information related to human social activities, namely, social information. On the basis of previous literature research, information alienation is summarized as follows: in the process of information production, dissemination, and use, the relationship between information producers, the main body of the information distributor, and the information object are unbalanced and the subject loses the ability of controlling the information. Therefore, the object in turn affects and controls the phenomenon of the subject [16].

In the social context, the process of information transmission is the process of human-computer interaction. The interpersonal dissemination of information determines the social characteristics of the information itself, and the alienation phenomenon produced by information is also closely related to social conditions. There are two main social reasons for the phenomenon of information alienation, as shown in Figure 1.

In recent years, there have been frequent occurrences of public opinion reversal and secondary disasters in many emergencies, which have brought a lot of inconvenience to social development and public life. Particularly, in the network communication environment, the information ecological environment is easily affected by the superposition of various factors, which leads to the proliferation of rumors, and the information originally produced and disseminated by humans in turn has a negative impact on social development and public life. Since many first-hand materials of emergencies are sent by netizens, the texts edited by netizens are often more emotional and have personal feelings. On the other hand, other netizens tend to take out of context and put their emotions first without knowing all the facts, which results in the alienation of information in the process of dissemination, which in turn controls public sentiment, misleads public opinion, breeds other events, disrupts the information ecology, and affects social stability [17, 18].

Some scholars have analyzed the difference between “information variation” and “information alienation” and pointed out that the word “variation” of information variation comes from the field of biology, which refers to the difference in variation between parents and children, as shown in Table 1. Information variation refers to a social phenomenon information dissemination process in which the concept of information transmission changes due to changes in related factors in the process of information dissemination. The information alienation studied in this paper is mainly to describe the relationship between people and information as producers and communicators, which arises in the process of information dissemination and utilization.

This model proposes a personalized push system model based on the memory-based collaborative filtering algorithm. The system is divided into three layers: application layer, service layer, and network layer. The system uses the application layer to obtain the user's browsing records and other personal information, transmits the information collected by the application layer to the data center of the service layer through the network layer, and uploads it to the dispatch center system through the distributed storage system. The user's interest information is generated by the algorithm in the dispatch center system, and the news is pushed to the user through the network layer. The whole model is divided into application layer, network layer, and service layer. The specific architecture is shown in Figure 2.

### 3.3. Intelligent Algorithm

Common intelligent algorithms include Tabu search (TS), simulated annealing (SA), genetic algorithm (GA), and ant colony algorithm (ACA) [19].

#### 3.3.1. Simulated Annealing Algorithm

The simulated annealing algorithm (SA) was first proposed in 1953. Until 1983, researchers applied the core idea of simulated annealing to complex combinatorial optimization problems and obtained good application results. Since then, the related application research of this algorithm has gradually enriched and expanded to many application fields. The algorithm is a stochastic optimization algorithm based on Monte-Carlo iterative solution strategy. The idea comes from the similarity between the physical solid-state cooling annealing process and many combinatorial optimization problems in mathematics. The annealing simulation algorithm starts from a given initial temperature and decreases the temperature parameter as it repeats. Combined with the probabilistic jumping ability of the algorithm, the solution of the objective function is randomly positioned in the feasible solution space of the problem, and the Metropolis criterion is used to determine whether a new solution will be accepted and repeat the process to gradually find the overall optimal solution to the problem [20, 21].

*(1) Mathematical Model*. If the energy of the particles is used to determine the state of the material, the Metropolis algorithm can describe the annealing process with a simple mathematical model.

Assuming that the energy of the material in state *a* is *E*(*a*), then the material goes from state *a* to state *b* at temperature *W* according to the following rules:

If *E*(*b*) ≤ *E*(*a*), accept the state to be transitioned.

If *E*(*b*) > *E*(*a*), then the following probability accepts state transitions:

(1) $$\begin{array}{c} e^{\left(E\left(a\right)-E\left(b\right)/\text{OW}\right)}. \end{array}$$

*O* is the Boltzmann constant in physics and *W* is the material temperature.

Currently, the probability that the material is in state *a* satisfies the Boltzmann distribution:

(2) $$\begin{array}{c} P_{T}\left(x=a\right)=\frac{e^{\left(E\left(a\right)/\text{OW}\right)}}{\sum_{b\in S}e^{\left(E\left(b\right)/\text{OW}\right)}}. \end{array}$$

*x* represents the random variable of the current state of the material, and *S* represents the state space set.

Obviously,

(3) $$\begin{array}{c} \underset{W⟶\infty }{\lim}\frac{e^{\left(E\left(a\right)/\text{OW}\right)}}{\sum_{b\in S}e^{-\left(E\left(b\right)/\text{OW}\right)}}=\frac{1}{\left|S\right|}. \end{array}$$

|*S*| denotes the number of states in the total *S*, when the temperature drops:

(4) $$\begin{array}{c} \underset{W⟶0}{\lim}\frac{e^{\left(E\left(a\right)-E_{\min}/\text{OW}\right)}}{\sum_{b\in S}e^{\left(E\left(b\right)-E_{\min}/\text{OW}\right)}}=\underset{W⟶0}{\lim}\frac{e^{\left(E\left(a\right)-E_{\min}/\text{OW}\right)}}{\sum_{b\in S_{\min}}e^{\left(E\left(b\right)-E_{\min}/\text{OW}\right)}+\sum_{b\in S_{\min}}e^{\left(E\left(b\right)-E_{\min}/\text{OW}\right)}}\\ =\underset{W\in 0}{\lim}\frac{e^{\left(E\left(a\right)-E_{\min}/\text{OW}\right)}}{\sum_{b\in S_{\min}}e^{\left(E\left(b\right)-E_{\min}/\text{OW}\right)}}=\left\{\begin{array}{c} \frac{1}{\left|S_{\min}\right|},ifb\in S_{\min i},\\ 0,\;\text{otherwise.} \end{array}\right) \end{array}$$

Among them, $E_{\min}=\underset{b\in S}{\min}E\left(b\right)$ and *S*_min_={*a|E*(*a*)=*E*_min_}.

*(2) Optimization Method*. The optimization function is as follows: *f* : *x*⟶*D*^+^, *x* ⟶ *S*, representing the feasible solution of the optimization problem, and *D*^+^={*y|y* ∈ *D*, *y* > 0}, S representing the domain of the function. *M*(*x*)⊆*S* represents a set of fields of *x*.

Given an initial temperature *W*_0_ and an initial solution *x*(0) of the optimization problem, *x*(0) creates the next solution *x* ′ ∈ *M*(*x*(0)), and whether *x*(1) accepts *x*′ as a new solution depends on the following probability:

(5) $$\begin{array}{c} P\left(x\left(0\right)⟶x^{\prime }\right)=\left\{\begin{array}{cc} 1, & \text{i}ff\left(x{}^{\prime }\right)<f\left(x\left(0\right)\right),\\ e^{\left(f\left(x^{\prime }\right)-f\left(x\left(0\right)\right)/W_{0}\right)}, & \text{otherwise.} \end{array}\right) \end{array}$$

If the function value of the resulting solution *x*′ is less than the function value of the previous solution, accept it as a new solution *x*(1)=*x*′. Otherwise, *e*^(*f*(*x*′) − *f*(*x*(0))/*W*_0_)^ accepts *x* ′'s new solution with probability. In general, for a specific temperature *W*_*a*_, a solution *x*(*o*) of the optimization problem can be created. The probability of being accepted *x*′ as the next new solution *x*(*o* + 1) is

(6) $$\begin{array}{c} P\left(x\left(o\right)⟶x^{\prime }\right)=\left\{\begin{array}{cc} 1, & \text{i}ff\left(x{}^{\prime }\right)<f\left(x\left(o\right)\right),\\ e^{\left(f\left(x^{\prime }\right)-f\left(x\left(o\right)\right)/W_{1}\right)}, & \text{otherwise.} \end{array}\right) \end{array}$$

The above equation shows that when the temperature drops too low, the material will enter the minimum energy state with high probability. Assuming that the problem we solve is an optimization problem of finding the minimum value, the annealing simulation optimization method is realized by applying the idea of annealing simulation to the physics of the optimization problem.

At the temperature of *W*_*a*_, after several transfers and lowering the temperature *W*_*a*_, *W*_*a*+1_ < *W*_*a*_ can be obtained.

Repeat the above process under *W*_*a*+1_.

*(3) Proving That the Algorithm Can Find the Global Optimal Solution*. Note that, in any *W*_*a*_ case, the obtained new state *x*(*o* + 1) is completely dependent on the previous state *x*(*o*) and possibly independent of the previous state *x*(0),…, *x*(*o* − 1), which is a Markov process. Using the Markov process to analyze the above simulated annealing step, the results show that the probability of any state *x*(*o*) generating *x* ′ is uniformly distributed over *M*(*x*(*o*)) and the probability of accepting the new state *x*′ satisfies formula (6). After a finite number of transformations, the distribution of equilibrium state *x*_*a*_ in temperature *W*_*a*_ is as follows:

(7) $$\begin{array}{c} W_{a}=\frac{e^{\left(f\left(x_{a}\right)/W\right)}}{\sum_{b\in S}e^{\left(f\left(x_{a}\right)/W_{a}\right)}}. \end{array}$$

When the temperature *W* will be 0, the distribution of *x*_*a*_ is

(8) $$\begin{array}{c} P_{a}^{*}=\left\{\begin{array}{cc} \frac{1}{\left|S_{\min}\right|}, & \text{if }\left(x_{a}\right)\in S_{\min},\\ 0, & \text{otherwise.} \end{array}\right) \end{array}$$

And

(9) $$\begin{array}{c} \sum_{x_{a}\in S_{\min}}P_{a}^{*}=1. \end{array}$$

This means that if the temperature drops too slowly and there are enough state transitions at each temperature to achieve thermal equilibrium at each temperature, the overall optimal solution will be found with probability 1. Therefore, it can be said that the annealing simulation algorithm is able to find the overall optimal solution.

#### 3.3.2. Genetic Algorithm

Genetic algorithm (GA) is an adaptive algorithm. Although there are many variations in the form of genetic algorithms in practical applications, these genetic algorithms have a common feature; that is, they imitate the natural selection, hybridization, and mutation mechanisms in the natural evolution process to complete the search for the optimal solution [22]. The evolution process of the genetic algorithm is shown in Figure 3.

Although the form of the optimization problem is different, the steps for applying the genetic algorithm to solve the optimization problem are basically the same, as shown in Figure 4.

The execution process of the genetic algorithm contains many random operations, so it is necessary to analyze its mathematical mechanism, leading to the following notation.

First, consider the result of the selection. In the standard genetic algorithm, the selection criterion is based on the principle of proportionality. Therefore, through the action of the *i*th selector, the expected value of the number of people who will continue to exist in the next generation is *n*(*f*_*a*_/∑*f*); then there is

(10) $$\begin{array}{c} \bar{f}\left(Z,r\right)=\frac{1}{n\left(Z,r\right)}\sum f_{a}. \end{array}$$

Then,

(11) $$\begin{array}{c} n\left(Z,r+1\right)=n\left(Z,r\right)\cdot \frac{\bar{f}\left(Z,r\right)}{f\left(r\right)}. \end{array}$$

The above formula shows that the effect of the selection operator will increase (decrease) the ability of a pattern above (below) the average to be applied across generations, improving quality.

Then, analyze the role of the crossover operator. This plan can obviously be maintained in the next generation if there is no intersection, or if the intersection point is beyond the character positions specified on the left and right ends of the figure. Therefore, the probability *W*_*s*_ that the *Z* mode will continue to exist in the next generation should satisfy

(12) $$\begin{array}{c} W_{s}\geq 1-W_{c}\cdot \frac{\varphi \left(Z\right)}{\left(L-1\right)}. \end{array}$$

Taking into account the effects of selection and crossover, there are

(13) $$\begin{array}{c} n\left(Z,r+1\right)\geq n\left(Z,r\right)\cdot \bar{f}\left(Z,r\right)\cdot \left[1-W_{c}\cdot \frac{\left(\varphi \left(Z\right)/\left(L-1\right)\right)}{\bar{f}\left(r\right)}\right]. \end{array}$$

Finally, the constant probability is 1 − *W*_*m*_ because *W*_*m*_ represents the probability that the mutation operator acts. If all the specified characters remain unchanged, the *Z* pattern can naturally continue to exist in the next generation; the probability (1 − *W*_*m*_)^*O*(*Z*)^, *Z*_*m*_ is usually not large; then under the action of the mutation operator the probability of *Z* continuing to exist is

(14) $$\begin{array}{c} {\left(1-W_{m}\right)}^{O\left(W\right)}\approx 1-W_{m}\cdot O\left(W\right). \end{array}$$

The probability that Z is unreserved is about *aW*_*m*_. So, taking into account the functions of selection, crossover, and mutation operators, we end up with

(15) $$\begin{array}{c} n\left(Z,r+1\right)\geq n\left(Z,r\right)\cdot \bar{f}\left(Z,r\right)\cdot \frac{\left[1-W_{c}\cdot \left(\varphi \left(Z\right)/L-1\right)\cdot W_{m}\right]}{\bar{f}\left(t\right)}. \end{array}$$

Specifically, if $\bar{f}\left(Z,r\right)=f\left(r\right)\left(1+c\right)$, *c* > 0 being constants, then

(16) $$\begin{array}{c} n\left(Z,r\right)=n\left(Z,r-1\right)\left(\Delta 1+c\right)=n\left(Z,O\right){\left(1+c\right)}^{r}. \end{array}$$

That is, functions with high average fitness grow exponentially in their ability of competing with other functions. However, high average conditions alone are not enough to guarantee high growth rates. When considering other impacts in detail, the definition of an operating model that requires good quality should be smaller in length and shorter in scope. High average suitability modes, low resolutions, and low order distances enable exponential growth in the number of solutions contained in generation after generation of group transmissions, which is the essence of the model theorem.

#### 3.3.3. Ant Colony Algorithm

Ant colony algorithm is a probabilistic algorithm for finding optimal paths. The observations suggest that ants leave secretions as they move and ants behind them make biased route choices based on the secretions that they leave behind. This is a positive feedback mechanism for learning information [23, 24]. Through this exchange of information, the shortest path to the searched food is described as

(17) $$\begin{array}{c} GA=\left(P\left(0\right),N,L,Q,U,P,F,Z\right). \end{array}$$

In formula (17), *P*(0) represents the initial group; *N* represents the overall number in the group; *L* represents the length of the binary; *U* represents the selection strategy. *G* represents the genetic operator; *P* represents the operation probability of *G*; *F* represents the fitness function; *Z* represents the termination rule.

The online performance is represented by the average from the first generation to the current generation, and *X*_*E*_(*U*) is defined as the linear performance of the *U* policy in environment *E*. *F*_*E*_(*Z*) is the objective function or the fitness function of the mean corresponding to time *Z* or environment *E* in the active generation; so

(18) $$\begin{array}{c} X_{E}\left(U\right)=\frac{1}{Z}\sum_{L}^{T}F_{E}\left(Z\right). \end{array}$$

Linear performance represents the average value of performance from the beginning of the algorithm to the current time period, reflecting the dynamic performance of the algorithm.

Offline performance is the cumulative average of the best performance, *X*_*E*_^*∗*^(*U*) is defined as the linear performance of *U* policy in environment *E*; then

(19) $$\begin{array}{c} X_{E}\left(U\right)=\frac{1}{Z}\sum_{L}^{Z}F_{E}^{*}\left(Z\right). \end{array}$$

Among them,

(20) $$\begin{array}{c} F_{E}^{*}\left(Z\right)=\text{BEST}\left(F_{E}^{\left(1\right)},F_{E}^{\left(2\right)},...,F_{E}^{\left(Z\right)}\right). \end{array}$$

The ant colony algorithm optimization process is actually controlled by three variables, namely, the state transition rule, the local pheromone update rule, and the general pheromone update rule.

The algorithm flow can be simply described as follows: each ant traverses all the cities according to the state transition rules and finds its own shortest path until all ants find their own solutions. Each time the repetition is completed, the pheromone on all routes is updated and the shortest route created after the repetition is recorded until the termination condition is met and the repetition ends [25]. In this process, the state transition probability can be defined as

(21) $$\begin{array}{c} P_{\text{AB}}^{K}\left(Z\right)=\frac{\varepsilon_{\text{AB}}^{i}\left(Z\right)\vartheta_{AB}^{j}\left(Z\right)}{\sum_{B=1}^{N}\varepsilon_{\text{AB}}^{i}\left(Z\right)\vartheta_{\text{AB}}^{j}}. \end{array}$$

Among them, *ϑ*_AB_ represents the visibility between the two locations *A* and *B*, *ε*_AB_ represents the concentration between the two locations, *i* represents the importance of the pheromone concentration between the two locations, and *j* represents the importance of the visibility between the two locations.

Using the memory list to record the list of cities that ant *K* has walked through, the formula can be updated as

(22) $$\begin{array}{c} \varepsilon_{\text{AB}}\left(Z+1\right)=w\varepsilon_{\text{AB}}\left(Z\right)+\Delta \varepsilon_{\text{AB}}\left(Z+1\right), \end{array}$$

(23) $$\begin{array}{c} \Delta \varepsilon_{\text{AB}}\left(Z+1\right)=\sum_{K=1}^{M}\Delta \varepsilon_{\text{AB}}^{K}\left(Z,Z+1\right), \end{array}$$

(24) $$\begin{array}{c} \Delta \varepsilon_{\text{AB}}^{K}\left(Z,Z+1\right)=\left\{\begin{array}{c} \frac{O}{L_{K}},\;\text{exit,}\\ 0. \end{array}\right) \end{array}$$

Δ*ε*_AB_^*K*^(*Z*, *Z*+1) is the amount of pheromone remaining on the path (*A*, *B*) when the *K*th ant moves at time (*Z*, *Z* + 1), and Δ*ε*_AB_(*T*, *T*+1) represents the amount of pheromone of all ants in this process. *O* represents the sum of all path pheromones, *L*_*K*_ is the total length of the path followed by the *k*th ant, and *w* is the decay factor of the pheromone trajectory. Figures 5 and 6 are the standard path construction diagram and the path construction diagram of the prospect strategy, respectively.

## 4. Control Experiment on the Problem of Media Information Alienation

### 4.1. Questionnaire Survey

This study conducted a questionnaire survey on 188 people, including 90 boys and 98 girls, selected from different age groups and different occupations, in order to make the data universal and authentic.

As scholars in various fields have conducted in-depth research on information pollution for many years, the concept and manifestation of information pollution have become stable. There are three forms of information pollution, namely, information garbage, information virus, and information infiltration. “Information garbage” also includes dirty information, useless information, and false information [26]. In resource sharing social media, the performance of “dirty information” is particularly obvious. Video sharing sites are more popular than pictures and music. In addition to the well-established Youku videos and Tudou videos, many video sharing sites have gradually emerged according to the characteristics of their respective video sites. Through the statistical survey of the questionnaire, the questionnaire raised two questions, “how often do you browse the filthy information” and “in which software you mainly browse (multiple choices);” the specific data is shown in Figure 7.

From the data in Figure 7(a), it can be seen that everyone will brush the dirty information. Among them, 12 people only brush it occasionally, accounting for 6.38%, and 40 people choose the general frequency, accounting for 21.28%. There are 89 people choose frequently, accounting for 47.34%, and 47 people who choose very frequently, accounting for 25.00%. It can be seen from this that filthy information has penetrated into the daily use of the Internet by the general public.

According to Figure 7(b), it can be seen that 98 people said that they would often swipe in music software, accounting for 52.13%, and 168 people chose to socialize, accounting for 89.36%. There are 86 people choose game software, accounting for 45.74%, 126 people choose shopping software, accounting for 67.02%, and 147 people choose video software, accounting for 78.19%. It can be seen from these data that all kinds of information have penetrated into all aspects of people's lives, and design software is the most commonly used software, so this may also be the reason for the most brushes. According to the survey, although such information is frequently swiped in social software, a large part of the reason comes from artificial transmission and frequent use.

### 4.2. Personalized Push Information Model

#### 4.2.1. Implementation of the Service Layer

*(1) Service Layer Design Principles*. The service layer is the core of the entire personalized recommendation model, and it is also the background of the network layer and the application layer, which stores the information in the entire system. The service layer includes the user information center, the algorithm recommendation layer, and the administrator system. The database of this model adopts MySQL, and the following principles are followed in the design of the database.

Data normalization: the relationship between the basic table and its fields should satisfy the third normal form (3NF) as far as possible. The third normal form achieves the best performance and integrity of the data and can properly eliminate redundancy.

Database field type specification: the data of a field should occupy as little space as possible, and the name should be concise and clear and named with English letters and natural numbers.

Data stability: ensure that the system will not crash due to a large amount of data. It can still ensure the speed efficiency of the operation when the amount of data is large.

*(2) User Information Center Design*. The user information center is a database for storing information, among which the user browsing information record table is the most important. This is used to store the user's personal browsing history, which type and which tag resource have been viewed, as shown in Table 2.

*(3) The Specific Design of the Administrator System*. Although the personalized push system all collects data autonomously and calculates similar user sets autonomously through algorithms, we still need administrators to manage the system so that users can have a better browsing experience, and the entire push model is more complete and more user-friendly. Therefore, in order to achieve the above goals, this paper joins the administrator system. The administrator can log in to the system anywhere with a network to manage the entire system. The main functions of the administrator system are the following.

Administrator login: the administrator is different from the user. The user logs in through the client, while the administrator logs in through the web page and distinguishes user categories according to personal information.

Feedback management: there is a feedback column on the client side, and administrators can watch and reply to users to improve the entire model and improve user browsing experience.

It has the highest authority; it can manage all users, with the authority to block, log out, unblock, etc.

Service layer management: it can manage the service layer, update the client, optimize the operation of the service layer, suspend or start the use of the service layer, and so on.

#### 4.2.2. Implementation of the Application Layer

*(1) Application Layer Design Principles*. The application layer is the App side for users to receive information. Users can browse to the information they want, and it is also responsible for collecting user data and personal information, providing all data sources for the personalized push model. The overall functions of the mobile phone information push system mainly include three main functional modules: push management, user management, and message management. It should follow these principles when designing the application layer.

Practicality, mobile terminal software, must firmly take the needs of users as the basic principle and push agricultural news on time, to achieve the purpose of convenient use; the operation interface is simple and clear, so that all agricultural workers can quickly get started, to achieve the purpose that anyone can use it.

Security ensures that the news pushed by the server can be successfully received and displayed and functions such as registration and modification of information can be used successfully, to reduce the failure of stalls and unexpected exits and to improve the App side.

*(2) User Management Design*. The user management and user registration diagram are shown in Figure 8.

*(3) Pushing Management and Message Management Design*. The specific design of push management and message management is shown in Figure 9.

Push management includes viewing unread and read messages. The push interval is set to meet the individual needs of users. Users can choose from instant push, every hour, every half day, every day, every three days, every six days, etc. The default interval for pushes is every hour.

Message management includes viewing favorite and subscribed messages and viewing feedback. Each message can be collected separately, and it can subscribe to such information. If there are any suggestions for the client, it can send them through feedback, and the feedback information can be viewed in the feedback view.

#### 4.2.3. Implementation of the Network Layer

The network layer is responsible for connecting the service layer and the application layer, uploading the user information including browsing records of the application layer to the service layer. This model uses OkHttp as the framework and JSON as the data transmission format, so the following principles are followed when designing the network layer:

Portability: using lightweight network protocols, the data transmitted is minimized and network traffic is reduced.

Reliability: the data received by the server is exactly the same as the data sent by the client, which can ensure that the data is not lost and error free.

Security: this takes appropriate encryption measures to ensure that data packets are not stolen by others, so as to protect the privacy of users.

### 4.3. Control of the Alienation of Information in Media Communication

#### 4.3.1. Control from the User Level

*(1) Improving the Information Literacy of Social Media Users*. The information literacy of social media users determines their ability of understanding and benefitting from information. Social media users vary greatly in their information literacy from as young as four or five to seventy or eighty years old. Many public homepages such as WeChat, Tencent, Sina, and Facebook have a lot of real-time news or professional domain knowledge. If the user's information literacy is low, it will exceed the user's ability of digesting. As a user who is both an information receiver and an information producer, such social media will do more harm than good. Consumers with high information literacy can accept and understand a large amount of information; otherwise, it will cause excess information. In addition, when the user's information literacy improves to a certain level, they will also realize the importance of their own information security, thus reducing the supervision of the social media environment and saving a certain amount of manpower and material resources.

The development of user information literacy can be divided into three stages: first, users need to have the ability of judging when information is needed. Although the information in the platform is updated in real time, it does not mean that it is needed at any time. Users should specify the time point when they need the information. Second, users need to know how to get the information. There are many types of social media platforms, striving to develop awareness of different types of media. Finally, users need to have the ability of using information rationally. It is a skill to effectively select what it need from a lot of information. After obtaining the required information, improving the efficiency of information use is the ultimate goal of cultivating users' information literacy.

*(2) Strengthening the Publicity and Education of Ethics, Morality, and Legal System*. As users of social media, when we enjoy the fast and convenient communication tools that this platform gives us and when we applaud the information transfer of music and video resource sharing, from the perspective of social media, low-quality and immoral Weibo spreading rumors, reprinting original articles on WeChat, and wanton abuse in forums not only violate the basic spirit of the “Outline of Citizen Morality,” but also violate the most basic ethical standards for users of social media platforms. It can be seen that the moral promotion of social media is necessary.

*(3) Improving the Copyright Awareness of the Original Content Published*. When looking at the similarities and differences between the Internet and social media, from the perspective of users, nearly 70% of users around the world are using social media. From the perspective of user usage time, the user's Internet usage time is only one-third of that of social media. It can be seen that the development trend of social media is pressing on the Internet step by step. Nowadays, the login of Sina Weibo, WeChat, blog, YouTube, and other social media requires registration as the user, and this registration process generally requires an e-mail or mobile phone number or even an ID number in some cases. This information should be protected as the user's privacy. Therefore, there is an urgent need to formulate comprehensive Internet user privacy protection regulations. As a service provider, it should be clearly stipulated that it is not allowed to collect and use users' information to obtain economic benefits; otherwise it should bear corresponding responsibilities and be punished accordingly. In addition to this, understanding real-time information, reading books, newspapers, and novels is another function of modern social media. The seemingly simple copyright requirement is what the original author has always called for. Wikipedia and Baidu, which have a large amount of information and a wide range of information, know that some distorted works and knowledge often appear, which not only confuses the user's audiovisual, but also violates the original work.

#### 4.3.2. Control from the Design Media Level

*(1) Control the Quality and Quantity of Information Resources*. Social media based on Web2.0 technology has a large amount of information resources, which is a major feature. The large amount of social media platforms that have not yet been developed will inevitably lead to difficult control and information pollution. Controlling the amount of information can avoid information redundancy, information excess, and information overload, so as to improve the utilization rate of information by users and avoid unnecessary waste. To control the amount of information, that is, the platform's control of information sources, establish a rigorous “information source control” mechanism. First, standardize information channels and then grasp information resources, striving to initially screen information at the source, so as to reduce the phenomenon of information alienation such as false information. Controlling the quality of information, that is, the platform's control of the ability of distinguishing information resources, on the basis of “quantity,” truly achieves “content supervision mechanism,” so as to provide users with a safe and clean social media platform.

*(2) Strengthening Information Security Technology*. Since ancient times, people have been trying various methods in order to gradually enhance their skills. The ancients improved their abilities through different media such as language, painting, and text. With the development of science and technology, human beings are faced with an increasing amount of information, and we can no longer rely on the brains and simple media to restrict behavior. Improving technology is the correct method. For users of social media, in addition to the fun and convenience brought by the application, when logging in to any social media, the most worrying thing is their own information security. In social media, information security issues have been common in recent years, and privacy leaks can be seen everywhere. Some information security issues require users to understand information security technology itself, and the other part requires social media service providers to further improve information security technology.

#### 4.33. Control from the Government Level

*(1) Establishing an Industry Supervision Association*. In the process of moving forward, any industry not only needs the law as the support for its correct development path, but also needs to assist and help the development of the industry in many aspects. At the same time, as the application of social media, the industry is developing rapidly and changing unpredictably. It is necessary to establish a supervision association for the industry, which can ensure real-time supervision when the law is not perfect and can also play an auxiliary role when the laws and regulations are improved.

In 2002, China promulgated the “China Internet Industry Self-discipline Convention,” which covered 31 contents. In order to promote the sound development of the industry and strengthen self-discipline, each province independently established the “Internet association.” However, with the expansion of the field of “social media,” there are some inapplicable clauses in the Internet self-regulation convention. Therefore, the author proposes establishing a separate “social media association” to promote the rapid and healthy development of social media. Different from the constraints of legal provisions, the writing time period of legal regulations is long, and it is difficult to integrate into the industry at one time; while the industry supervision association is more flexible, it is easy to change its thinking according to the current social media development situation and can make real-time adjustments. Thirdly, the monitoring association not only monitors whether the social media platform is used legally, but also protects the users of the social media platform at another level. It is like a nexus that, along with the government's legal oversight of social media, also urges social media itself to move in the right direction. Because industry supervision associations are not affiliated to government agencies but are spontaneously initiated by the people, they are more mobile and flexible.

*(2) Laws and Regulations for Establishing Social Media*. The “constitution” is China's basic law. Since the development of social media, the application of social media has long been regulated in accordance with the rules and regulations of the “Administrative Measures for Internet Information Services” promulgated in 2000. But social media has moved forward at an alarming rate, and many regulations are now a thing of the past and still need to be refined and adjusted. The only management methods cannot fully keep up with the times. It is necessary to clarify the laws and regulations of social media at various stages and to explain in detail from the establishment, application, and punishment methods of illegal and criminal social media. The boundaries between “social media” and “Internet” should be clearly defined, and the concept of “noncommercial Internet information services” should be clearly defined.

## 5. Discussion

First of all, through the study of relevant knowledge points of literature works, this paper initially masters the relevant basic knowledge and analyzes how to research the alienation technology control of push information based on intelligent algorithms. This paper expounds the concept and algorithm of intelligent algorithm simulated annealing algorithm, studies genetic algorithm, explores ant colony algorithm, and analyzes the applicability of alienation technology control in pushing information through experiments.

The alienation of information will have a huge impact on the normal life of government departments and the public, and the credibility of the government will decline. The public's demand for information on emergencies and the supply of government information are unbalanced, which makes rumors enter the information transmission channels, mix them with falsehoods, and confuse the truth. The decline of the government's credibility has caused the public to be reluctant to give the official a waiting period and reduce the social trust among the public. The spread of rumors and fake videos confuses public opinion and misleads public sentiment. People are troubled by their own emotions, causing rumors to spread. While consuming public resources, it reduces the trust between people, aggravates social conflicts, and affects the construction of social spiritual civilization. By effectively improving the media literacy of citizens and accelerating the formation of a correct cognitive framework, we can reconstruct the social trust system and build a benign information ecological environment [27–29].

Through the experimental analysis in this paper, we can see that the control of the alienation of media dissemination information is not enough and it needs to be controlled from multiple aspects. By improving the information literacy of social media users, strengthening the publicity and education of ethics, morality, and legal system, enhancing the awareness of the copyright of the original published content, controlling the quality and quantity of information resources, and strengthening the information security technology, the government establishes social media laws and regulations through the establishment of industry supervision associations; in this way, the problem of information alienation will be properly solved.

## 6. Conclusions

In the new media environment, a new communication ecology and multiple public opinion patterns have been formed. The dissemination of information has the characteristics of the new era, such as the suddenness, urgency, and extensive influence of emergencies. This makes it easy to be alienated by man-made and environmental influences in the process of information dissemination, which has a negative impact on the truth of events and social stability. The ongoing “news reversal” and “public opinion reversal” incidents invisibly eliminate social trust, weaken the credibility of the media, and are not conducive to the relationship between leaders and the masses and the construction and maintenance of public relations. With the rapid development of new media technology, how to distinguish the authenticity of information and look at things objectively and rationally in the information age with the speed of light development is worthy of public reflection and learning. For the relevant government departments, it is the focus of today's work to be a transparent, open, and service-oriented government without official pretensions and to form a positive interaction with the public. Both new and old media should clarify their own responsibilities, strengthen industry self-discipline, and be a good watcher of the society in the dissemination of information.

## Figures and Tables

**Figure 1:** Social causes of information alienation.

**Figure 2:** Model construction diagram.

**Figure 3:** Schematic diagram of genetic algorithm evolution.

**Figure 4:** Schematic diagram of applying genetic algorithm to solve the problem.

**Figure 5:** Standard path construction.

**Figure 6:** Path construction for the outlook strategy.

**Figure 7:** Propagation data for dirty information. (a) Frequency of viewing obscene information. (b) Main website penetration rate.

**Figure 8:** User management specific design. (a) User management diagram. (b) User registration diagram.

**Figure 9:** The specific design of push management and message management. (a) Push management diagram. (b) Message management diagram.

**Table 1:** Discrimination of the concepts of information alienation and information variation.

	Information alienation	Information variation
Core significance	The relationship between people and information	Attribute of information itself
Generation time	When information is highly active	With the development of human life
Coverage space	Certain events	Every corner
Research characteristics	Focus on conclusion	Dynamic process
Discipline	Informatics, information science	Journalism and communication

**Table 2:** User browsing information record table.

Character name	Character type	Character description
User_ id	Varchar	User ID
User_ name	Varchar	Username
User_ sex	Int	User gender
Category_ jid	Int	Browsing type
Label_ id	Int	Browse tab
User_ browse times	Varchar	Views
Earliest browsing	Date	See this first
Recently browse	Date	Recently watched this time

## Data Availability

The data that support the findings of this study are available from the corresponding author upon reasonable request.
